The article "Early Warning of Enterprise Financial Risk Based on Decision Tree Algorithm" was published in 2022. Journal: Comput Intell Neurosci.

# Early Warning of Enterprise Financial Risk Based on Decision Tree Algorithm

**DOI:** 10.1155/2022/9182099

**Published:** 2022-07-14

**Authors:** Sen Hong, Han Wu, Xiujuan Xu, Wei Xiong

**Affiliations:** Jiangxi University of Engineering, Xinyu 338029, China

## Abstract

To improve enterprise financial early warning, we propose an algorithm based on a decision tree. According to the shortcomings and defects of the classical algorithm and the traditional decision tree algorithm, in the ordinary decision tree improved algorithm based on PCA, there is a problem that the representativeness of the data after dimensionality reduction processing are not high, resulting in the fact that the accuracy of the algorithm can be improved slightly after multiple data runs. Based on the classical algorithm, attribute eigenvalues before classification are extracted twice, and the amount of data to be classified is calculated. That is, the most important attributes of the original data are selected. After the subtree is established, the dimension reduction and merging selection of the data are performed, and the improved algorithm is verified by using three data sets in the UCI database. The results show that the average accuracy in the three datasets is 94.6%, which is improved by 1.6% and 0.6% for the traditional classical algorithm and the ordinary PCA decision tree optimization algorithm, respectively. PCA-based decision tree algorithms can improve the accuracy of the results to some extent, which is of practical importance. In the future, a classic algorithm improved for secondary modeling will be used to obtain a more efficient decision tree model. The decision tree algorithm has been proven to recognize an early warning of an enterprise's financial risks, which enhances the effectiveness of an enterprise's early financial warning.

## 1. Introduction

In the post-financial crisis period, enterprises are in an unpredictable external environment, and different forms of risks emerge one after another. The survival and development of enterprises are inseparable from the external environment. At the same time, the uncertainty of the external environment has a nonnegligible impact on the daily operation of enterprises. Additionally, the negligence or change of any link in the daily operation of enterprises, if not identified and controlled in time, is likely to lead to financial risks. With the increasing degree of economic globalization, the complex and changeable market environment makes enterprises face more financial risks different from the past [1]. Additionally, through the tree algorithm, the problems in decision-making and control in enterprise operation and management activities, such as the difficult recovery of accounts receivable, improper authority setting, wrong financing decision-making, and investment decision-making, will lead to financial risks and bring huge economic losses to the enterprise if they cannot be identified and handled in time. Under the background of the contemporary market economy, any enterprise is in an extremely complex living environment and cannot obtain all the information to make it grow, which determines that the enterprise will face certain financial risks. Recently, the outbreak of the financial crisis has shifted the focus of attention to the risk management of enterprises, especially the importance of financial risk management. At present, in the daily operation and management of enterprises, financial risk management is still ignored by most Chinese enterprises, and financial risk still exists in enterprises. For example, the setting of financial control right is unreasonable, and the financial governance structure is imperfect [2]. The financial control mode lags, and the financial early warning analysis and control mechanism are not perfect. The concept of financial risk management is backward, and the concept of risk value is insufficient. Internal audit exists in name only, and internal financial supervision is lacking. Recently, from the various financial failure cases of Chinese enterprises, people have deeply realized that further research on enterprise financial risk management has a theoretical and practical significance that cannot be ignored. This kind of information is defined as an internal report. The internal report provides managers at different levels with the information they need for business decision-making and control, to timely adjust the business management strategy and make corresponding decisions. Additionally, compared with the external reports, not only do the internal reports have the functions of precontrol and in-process control after reporting and presentation but also attract more and more attention from enterprise management. However, compared with the development of financial accounting, the development and attention of management accounting are still backward. At the same time, the theory of management accounting is divorced from practice, and a complete theoretical framework that can guide and apply to management accounting practice has not been formed [3, 4]. Among them, there is less research on the theory and system of internal reports, and there is no unified concept of internal reports. Currently, a few internal reports in enterprises are mostly prepared for the final completion of external reports, which cannot give full play to the value of internal reports.

The main goal of this paper is to optimize the decision tree algorithm and apply it to enterprise cost control. Therefore, the basic technology and theory based on this research mainly include data mining technology and decision tree algorithm. Common data mining technologies include the following main contents in the implementation process. From front to back, these contents are to ask questions according to needs, make necessary data preparation, preprocess massive data, build data mining models, and evaluate and explain the models. The model system of the whole data mining is shown in Figure 1.

## 2. Related Work

Kumar and Ragava Reddy sorted out and analyzed the reasons for the operation failure of small and medium-sized enterprises in Finland with reference to the evaluation method of Bank of America on the operation and financial status of small and medium-sized enterprises [5]. The research found that the lack of management ability of middle-level managers, the lack of information provided by the accounting system, and the attitude of enterprises towards employees have an important impact on the operation failure of enterprises. This research result provides a new direction for evaluating the financial and operating status of enterprises. Xu et al. used a variety of mixed financial risk early warning models, that is, different combinations of multivariable discriminant analysis, logistic regression, and BP neural network methods to conduct an empirical analysis of the sample data. Through research, it was found that the prediction accuracy of the mixed early warning model was significantly higher than that of a single early warning model [6]. Clarin conducted in-depth research on the safety management problems and countermeasures of foreign students in colleges and universities, expounded on the importance of early warning mechanisms, and established early warning mechanisms for emergencies, cultural conflicts, accidental injuries, and other problems endangering the personal safety of foreign students during their stay in China. The early warning mechanism can discover the causes of contradictions in advance, and managers can take measures in advance to reduce the impact scope of safety events and even avoid the occurrence of safety events, so as to achieve the transformation from remedying the occurrence of events to early warning to avoid the occurrence of events [7]. When exploring the management strategy of foreign students in China in the new era, Hammed and Jumoke mentioned the need to establish a prevention mechanism for emergencies of foreign students [8, 9]. Hassan et al. conducted an in-depth study on the construction of the emergency early warning and prevention mechanism for foreign students in China and expounded the necessity of the safety early warning mechanism for foreign students. In terms of the purpose and effect of safety event management, “plan ahead” is far better than “make up for the lost.” Li et al. was the first scholar to use regression analysis to study financial risk early warning. The emergence of this research made discriminant analysis replaced by regression analysis and became the mainstream method in the field of financial crisis early warning in the 1980s [10]. Zhang et al. referring to the evaluation method of Bank of America on the operation and financial status of small and medium-sized enterprises, sorted, and analyzed the reasons for the operation failure of small and medium-sized enterprises in Finland. The research found that the lack of management ability of middle-level managers, the lack of information provided by the accounting system, and the attitude of enterprises towards waiting for employees have an important impact on the operation failure of enterprises. This research result provides a new direction for evaluating the financial and operating status of enterprises [11]. Bian and Wang empirically analyzed the sample data by using a variety of mixed financial risk early warning models, that is, different combinations of multivariate discriminant analysis, logistic regression, and neural network methods. The research found that the prediction accuracy of the mixed early warning model is significantly higher than that of a single early warning model [12]. When conducting univariate analysis on the financial status of sample enterprises, Oujdi et al. selected a financial ratio, including asset liability ratio, return on net assets, return on total assets, and current ratio. The research results show that the asset liability ratio and current ratio have the lowest misjudgment rate on the financial status [13, 14]. Nguyen et al. studied the financial risk early warning model based on fuzzy neural network, selected variables from three alternative financial indicators through stepwise regression method, and finally locked the indicators of long-term liabilities, shareholders' equity, profit growth rate, current ratio, total working capital assets, asset turnover, and asset return as the final analysis variables.

Based on existing research, a tree-based algorithm is being developed. Algorithm improvement depends on the inadequacy of classical algorithms and always deciding tree algorithms. Data research has shown that there are many ways to select the determination of classical algorithms. Therefore, this paper presents an algorithm for optimizing tree decisions based on PCA. In an algorithm for improving PCA-based decision making, the problem is that the representation data is not very high after the reduction in size. As a result, the accuracy of the algorithm improves slightly after data recovery. According to the classical algorithm, this dataset counts the value of the identity of the behavior before the two groups and counts how much data to divide, for example, selecting the most important objects of the data in old papers, creating a subtree, reducing the cost of data, and growing and consolidating information. The development algorithm has been validated using our dataset in the UCI database.

## 3. Method

Some research on specific issues requires the collection of data and the use of data, and classical procedures for this data often have many differences, and the relationship between differences are difficult to find intuitively. However, there are several factors that often play an important role in the integration of classical algorithms. Therefore, we need to pay attention to the hidden connection and learn more about the relationship of the relationship matrix of the first difference in the data structure of the classical algorithm or internal structure of the covariance matrix and identify the algorithm of linear combinations of the first variables of the data algorithm. The first classical algorithm, obtained by many incomplete, we call it the main component. The classical algorithm generally maintains the following relationships between the main components and the base components obtained after calculating the original variables.

1. The main idea is the composition of the source material.
2. The number of critical points is less than the number of original objects.
3. Most of the information contained in the initial variables is stored in each principle.
4. Independence of the two priorities is established. After the analysis, we can see the key points from the differences of the first ones that contain the basic characteristics, so that when we are faced with a lot of data, we can reach a numerical analysis and then study and understand the relationship between the initial differences. The internal rules of product research and the results are studied at a deeper level. The steps of principal component analysis are as follows: let the thing we want to study contain *P* indexes, expressed as *x*_1_.*x*_2_ … *x*_*p*_, and the *p*-dimensional random vector that can be formed by this index is (*x*_1_.*x*_2_ … *x*_*p*_). Let the mean of random vector *X* be *u* and the covariance matrix be e [15, 16]. Next, we perform linear transformation on *X*. after this step, we can get a new comprehensive variable *Y*. In other words, the new comprehensive variable can be described linearly by the original variable; that is, it meets the following requirements:

(1) $$\begin{array}{c} y_{1}=\mu_{11}x_{1}+\mu_{12}x_{2}+\cdots +\mu_{1p}x_{p},\\ y_{2}=\mu_{21}x_{1}+\mu_{22}x_{2}+\cdots +\mu_{2p}x_{p},\\ y_{p}=\mu_{p1}x+\mu_{p2}+\cdots +\mu_{pp}x_{p}. \end{array}$$

Because we can make the above linear changes to the original variables, the statistical characteristics of the comprehensive variable *Y* will change with different linear transformations. Therefore, to obtain better results, the variance of *y*_*i*_=*μ*_*i*_^,^*x* should be kept as large as possible, and each y_*i*_ should be independent, because

(2) $$\begin{array}{c} \mathrm{var}\left(Y_{i}\right)=\mathrm{var}\mu_{i}^{,}x=\mu_{i}^{,}\sum \mu_{i}. \end{array}$$

Given any constant C, you get

(3) $$\begin{array}{c} \mathrm{var}\left(c\mu_{i}^{,}x\right)=c\mu_{i}^{,}\sum \mu_{i}c=c^{2}\mu_{i}^{,}\sum \mu i. \end{array}$$

Therefore, if *P* is not limited, var(*Y*_*i*_) can be increased at will, which makes the problem meaningless [17]. Linear transformation constraints need to be carried out under the following principles:

(1) (4) $$\begin{array}{c} \mu_{i}^{,}\mu_{i}=1. \end{array}$$
The following is obtained:
  (5) $$\begin{array}{c} \mu_{21}+\mu_{22}+\cdots +\mu_{2p}=1\left(i=1,2\ldots ,p\right). \end{array}$$
(2) *Y*_*i*_ and *Y*_j_ are not related to each other (*i* ≠ j, *i*, *j*=1,2 …, *p*).
(3) *Y*_1_ is the maximum term of the variance obtained in the linear combination of *X*_1_, *X*_2_,…, *X*_*p*_ satisfying principle 1.

*Y*_2_ is the largest term of variance among all linear combinations of *X*_1_, *X*_2_,…, *X*_*p*_ independent of *Y*_1_; …*Y*_*p*_ is the largest term of variance among all linear combinations of *X*_1_, *X*_2_,…, *X*_*p*_ not related to *Y*_1,_, *Y*_2_,…*Y*_*P*−1_.

The comprehensive variable *Y*_1,_, *Y*_2_,…*Y*_*P*_ determined under the previously mentioned three principles is called the 1,2,…, *p*-th principal component of the original variable, and the proportion of each comprehensive variable in all variance sum is decreasing. In our research, we usually only select the first few components, to simplify the model.

In the traditional ID3 algorithm, the attributes of different individuals are different at the specific value level, and the subset constructed by the algorithm is the training set divided based on this different value. Therefore, the number of subsets finally constructed by ID3 algorithm is the same as the number of types of individual attributes. On this basis, when building the decision tree, the subset corresponds to the branches of the decision tree, and the end points of these branches become leaf nodes, resulting in corresponding decision rules [18]. In this case, if there are too many kinds of attribute values, it will obviously directly increase the leaf nodes, decision paths and finally formed decision rules of the decision tree. That is, it will increase the overall scale of the decision tree, and even lead to the multivalue tendency of decision attributes, resulting in the low accuracy of decision rules. Then, the optimization of ID3 algorithm proposed in this paper is to solve such problems. The specific optimization ideas are as follows.

1. Select training to determine classification attribute AK.
2. Establish a node *n*.
3. If the data under consideration are of the same category, *n* is the decision tree leaf and the class is the leaf.
4. If there are no other properties that can be analyzed in the current data under consideration, *n* is also a leaf at this time, and the classification of leaves is marked according to the principle of minority obedience to the majority.
5. Otherwise, select the average value of the attribute *n* along the test node with the best expected value of the attribute.

The algorithm is initially based on the original ID3 decision tree algorithm. The main idea is as follows.

Step 1: select the file, first compress the file using PCA algorithm, and select the key operations. During this time, the data is compressed using the PCA algorithm. Currently, there are many differences in the process of tree design decisions, and the relationship between the differences shows that there are many controls. We use this data to analyze and study the internal structure of the bond matrix or the covariance matrix of the original data exchange. For example, coefficient matrix can be created as follows [19].
Step 2: initialize the data we need to process to construct a complete data matrix. *X*_*m∗n*_, *m* represents the number of records, and *n* represents the dimension of data records.
Step 3: for data standardization, the average of the data is 0, and the standard deviation is 1. That is, data with different dimensions is entered into the same matrix. The mathematical models for normalizing data are as follows:
  (6) $$\begin{array}{c} Z\left(X\right)=\frac{x-\bar{x}}{s\left(x\right)},\\ \frac{x-\bar{x}}{s\left(x\right)}=\frac{x-\bar{x}}{\sqrt{{\left(x-\bar{x}\right)}^{2}/n}}. \end{array}$$
Step 4: solve the differences between the matrix files. The purpose of problem solving is to measure the relationship between two differences, and the models are as follows:

(7) $$\begin{array}{c} \mathrm{cov}\left(x,y\right)=\frac{\sum_{i=1}^{n}\left(X_{i}-\bar{x}\right)\left(Y_{i}-\bar{Y}\right)}{n-1}. \end{array}$$

When we encounter an *n*-dimensional matrix data, we can obtain the difference between the two datasets. Thus, this *n*-dimensional data can be obtained from the *n∗n* covariance matrix [20].

(8) $$\begin{array}{c} \mathrm{cov}\left(X_{n*n}\right)=\left(C_{ij},C_{ij}=\mathrm{cov}\left(\dim_{i},\dim_{j}\right)\right). \end{array}$$

If *X*_*i*_ represents the *i*th attribute of the matrix, it can be expressed as follows:

(9) $$\begin{array}{c} Coeff=\left[\begin{array}{ccc} \mathrm{cov}\left(x_{1},x_{i}\right) & \ldots & \mathrm{cov}\left(x_{1}x_{n}\right)\\ \ldots & \ldots & \ldots \\ \mathrm{cov}\left(x_{n},x_{1}\right) & \ldots & \mathrm{cov}\left(x_{n}x_{n}\right) \end{array}\right]. \end{array}$$

Then, we use the linear combination of the original variables to get some comprehensive indicators, which is what we call the principal component.

## 4. Experimental Results and Discussion

To verify the optimization algorithm, the author selected the data from UCI machine learning database for the experiment. The first selected is the wine dataset, which contains 178 samples and 13 attributes. After substituting into the original ID3 algorithm and the operation comparison of the optimization algorithm, as shown in Figure 2.

In Figure 2, the original ID3 algorithm had five conflicts and only two conflicts after improvements, confirming that the optimization accuracy was higher than the original algorithm [21]. Additionally, experiments were performed on adult data and vehicle datasets and compared with the same PCA as the ID3 algorithm. The results are shown in Figure 3.

In Figure 3, in the comparison data, the algorithm is more accurate than the original ID3 algorithm and PCA hybrid algorithm. There is reason to believe that the algorithm has improved. For clarity, the results are shown in Figure 4.

After double compression of the test samples, the accuracy of the optimization was improved to some extent. The accuracy of the optimization algorithm is 2.2% higher than that of the traditional ID3 algorithm and 1% higher than that of the traditional PCA sheep algorithm. The accuracy of the adult data is 1.1% higher than the standard ID3 standard and 0.6% higher than the PCA melting algorithm. The accuracy of the optimization algorithm of vehicle dataset is 1.4% higher than the traditional ID3 algorithm and 0.1% higher than the PCA integration algorithm. Additionally, two data mining algorithms, KNN and naïve Bayes, were tested and integrated into the adult data set for comparison and use. Of these, the accuracy of the KNN algorithm is 87.5% and the accuracy of the Naive Bayes algorithm is 93.75%, which is lower than the performance of this form factor. The algorithms described in this paper have been proven in practice to be practical. The new algorithm, optimized for the ID3 algorithm, has the following advantages.

1. The optimization algorithm effectively solves the problem of multivalue tendency of traditional ID3 algorithm in decision attributes. That is, through principal component analysis, select more representative decision attributes, so as to avoid the multivalue tendency after the calculation of decision attribute information entropy and the reduction of decision attributes, which will inevitably reduce the overall time of decision tree modeling and improve the efficiency of decision tree modeling.
2. After the establishment of subtree, PCA algorithm is used to compress again, and the merged branches are marked with nodes, and then, they are continuously split, which not only effectively avoids the limitations of first pruning but also makes effective use of all datasets. To further verify the advantages of the optimization algorithm, this paper is also based on the dataset of an agricultural material enterprise in the previous paper. In Windows 10 operating system, Python is used to rewrite the optimization algorithm, and the rewritten algorithm is simulated. That is, the secondary modeling of the cost control of an agricultural material enterprise is implemented to obtain a new decision tree model as shown in Figure 5.

Additionally, according to the new decision tree, some rules related to the cost control decision of an enterprise can be obtained. These rules are different from the rules obtained by ID3 algorithm. The specific rules are as follows.

1. If main business cost control = excellent, then cost control = excellent.
2. If main business cost control = qualified and management cost control = excellent, then cost control = excellent.
3. If main business cost control = qualified and management cost control = qualified and sales cost control = unqualified, then cost control = unqualified.

From the previously mentioned experimental results, we can find that when using the improved algorithm in this paper, only three cost items are retained through PCA algorithm. To include the production cost for analysis, the overall tree view is more streamlined [22]. Moreover, according to the evaluation results after the completion of decision tree modeling, the accuracy of decision tree modeling using optimization algorithm is higher, up to 95.1%. The modeling time is shorter, which is 8.2 seconds. Additionally, we also substituted the data into the ordinary PCA fusion algorithm, and its accuracy rate reached 94.2, but the time spent is less than the optimization algorithm in this paper, which is 7.8 seconds.

According to the decision tree modeling of the traditional ID3 algorithm and the modeling results of the new optimized algorithm, there is no small difference between them. From the perspective of decision tree modeling time, the newly optimized algorithm improves the accuracy of the algorithm to a certain extent due to the compression and dimensionality reduction of decision attributes, and the operation time is also less than that of the original ID3 algorithm. The comparison results of the algorithm before and after optimization in decision tree modeling time are shown in Figure 6. There is no doubt that the optimized algorithm is faster in decision tree modeling, and the modeling time is 4.4 seconds shorter than the traditional ID3 algorithm.

Additionally, from the accuracy level of decision tree model, there are also differences in ID3 algorithm before and after optimization. The accuracy of modeling is compared, and the results are shown in Figure 7.

According to Figure 6, it is not difficult to find that the optimized algorithm has higher accuracy in decision tree modeling than the traditional ID3 algorithm and ordinary PCA combined algorithm, which shows that the optimized algorithm is more accurate and can be used in decision tree modeling. In other words, after comparing ID3 algorithm with the optimization algorithm in this paper, the specific comparison data in modeling time, decision tree size, prediction rules, and accuracy can be obtained, as shown in Figure 8.

We can see that the optimized algorithm has obvious advantages in terms of modeling time, total number of nodes, number of leaf nodes and number of decision rules, which is more practical for the construction of enterprise cost control decision tree.

In early warning, we should first make a preliminary analysis of the company's annual reports in recent years to teenagers, judge which link of the current company's financial situation is in the early warning chain, and then determine the early warning path and early warning target. Then, according to the early warning link, determine the index system, select and calculate relevant financial indicators, make up for the missing data, and then standardize. The comprehensive indicators are calculated using factor analysis and other methods. Finally, several early warning models are used to warn the financial situation in the next period.

Through the traditional multipurpose regression model for financial risk early warning, the dependent variable of the general multiple linear regression model is a continuous variable. When the dependent variable is a binary value or variable, if the classical regression model is established, the model is likely to no longer be effective. Therefore, for the data with dependent variable the regression model should be used, and its function form is as follows.

(10) $$\begin{array}{c} y=f\left(x\right)=\frac{1}{1+e^{-x}}=\frac{e^{x}}{1+e^{x}}. \end{array}$$

Let Π represent the probability of *y* = 1, which is recorded as *P*(*y* = 1) = Π, and the probability of *y* = 0 is *p* (*y* = 0) 1 − Π. It is assumed that there are *n* explanatory variables *x*_1_, *x*_2_ … *x*_*n*_, , which are recorded as (*x*_1_, *x*_2_ … *x*_*n*_,)^,^ by vector *X*. different from the linear model. The logistic model does not study the relationship between the dependent variable value and the explanatory variable, but the relationship between the dependent variable value probability Π and the explanatory variable [23]. In fact, the relationship between probability Π and explanatory variables is not a simple linear relationship, but an “*s*” curve. At this time, the logical curve model is expressed as

(11) $$\begin{array}{c} \pi =p\left(y=1|X\right)=\frac{\exp\left(\beta_{0}+\beta_{1}x_{1}+\cdots +\beta_{n}x_{n}\right)}{1+\exp\left(\beta_{0}+\beta_{1}x_{1}+\cdots +\beta_{n}x_{n}\right)}=\frac{\exp\left(X\beta \right)}{1+\exp\left(X\beta \right)}. \end{array}$$

Logit transforms the previously mentioned formula to obtain

(12) $$\begin{array}{c} \text{Logit}\left(y\right)=In\left(\frac{\pi }{1-\pi }\right)=\beta_{0}+\beta_{1}x_{1}+\cdots +\beta_{n}x_{n}=X\beta . \end{array}$$

The previously mentioned formula is the logistic regression model, in which *β*_0_, *β*_1_ … *β*_*n*_ is the parameter to be estimated.

*β*_0_, *β*_1_ … *β*_*n*_ can be estimated by maximum likelihood and solved by Newton-Raphson iteration.

For *m* samples, there are *P*=(*y*_*i*_=1)=*π*_*i*_ and *P*=(*y*_*i*_=0)=1 − *π*_*i*_, where *i* = 1,2,…, *m*. Then, the joint probability density function of *y*_*i*_ is

(13) $$\begin{array}{c} P\left(y_{i}\right)=\pi_{i}^{yi}{\left(1-\pi_{i}\right)}^{1-yi},y_{i}=0,1. \end{array}$$

The detection rate is defined as the possibility of risk samples found by the early warning model. The detection rate focuses on whether it can be found effectively. The definition accuracy rate is the accuracy of early warning discrimination after the early warning results come out. The accuracy rate focuses on whether the early warning results are accurate. Calculate the risk value of training samples according to the early warning model and verify the early warning effect of the model. The results are summarized in Table 1.

In terms of detection ability, there are training samples marked as in the original data and the number of successful predictions by the early warning model. Among them, there are samples that are misjudged as normal, and the detection rate of risk samples is as high as 76.1%. There are samples marked as in the original data, and there are samples that are successfully predicted, among which there are samples that are misjudged as risk samples, and the detection rate of normal samples is 68.2%, nearly 70%, and the recognition rate of normal samples is slightly low. The average detection rate of the model is 72.1%. The overall detection effect of the established logistic early warning model is good, which can basically be used for actual early warning.

The probability of early warning is 72.5%, while the probability of accurate early warning is 29.5% when the sample is normal, and the probability of accurate early warning is 3.5%. The detection rate and accuracy of logistic early warning model are equivalent.

Taking the total early warning effect as the arithmetic mean of average detection rate and average accuracy, the total early warning effect of logistic model is 72.2%.

## 5. Conclusion

This paper studies the specific application of decision tree algorithm in enterprise cost control. The application of data mining technology first needs to clarify the data mining requirements, which is the prerequisite before each data mining task is established. Only by clarifying the data mining requirements, can we further determine what kind of data to choose and what algorithm to use for data mining, to make the realization goal of data mining more targeted. From the previously mentioned experimental results, we can find that when using the improved algorithm in this paper, only three cost items are retained through PCA algorithm. To include the production cost for analysis, the overall tree view is more streamlined. Moreover, according to the evaluation results after the decision tree modeling is completed, the accuracy of decision tree modeling using the optimization algorithm is higher, up to 95.1%, and the modeling time is shorter, 8.2 seconds. Additionally, we also substituted the data into the ordinary PCA fusion algorithm, and its accuracy reaches 94.2, but the time spent is less than the optimization algorithm in this paper, which is 7.8 seconds.

## Figures and Tables

**Figure 1:** Basic architecture of data mining.

**Figure 2:** Comparison of results of wine dataset. (a) Results under the original ID3 algorithm. (b) Results of optimized algorithm.

**Figure 3:** Comparison of algorithm accuracy.

**Figure 4:** Comparison of accuracy of algorithm results.

**Figure 5:** Decision tree of agricultural materials enterprises obtained by optimization algorithm.

**Figure 6:** Comparison of algorithm decision tree modeling time before and after optimization.

**Figure 7:** Comparison of accuracy of algorithm decision tree before and after optimization.

**Figure 8:** Comparison and summary of algorithms before and after optimization.

**Table 1:** Effect of logistic model.

		Prediction results		Detection rate	Average detection rate
0	1				

Original mark	0	299	94	76.1%	72.1%
	1	125	268	68.2%	
Accuracy		70.5%	74.0%	Total early warning effect	
Average accuracy		72.3%		72.2%	

## Data Availability

The data used to support the findings of this study are included within the article.
